# Effect of Salvia Miltiorrhiza Polyphenolic Acid Injection on Improving Limb Use and Cognitive Impairment in Patients with Acute Stroke

**DOI:** 10.1155/2022/1481294

**Published:** 2022-08-09

**Authors:** Shan Cong, Chunxue Dong, Yujiao Hu, Chunying Wang, Bingquan Zhang, Nan Li

**Affiliations:** ^1^The Second Affiliated Hospital of Qiqihar Medical University, Clinical Pharmacy, China; ^2^The Second Affiliated Hospital of Qiqihar Medical University, Department of Rehabilitation Medicine, China; ^3^Department of Neurology, The Second Affiliated Hospital of Qiqihar Medical University, China; ^4^The Second Affiliated Hospital of Qiqihar Medical University, China; ^5^The Second Affiliated Hospital of Qiqihar Medical University, Pharmacy Intravenous Admixture Services, China

## Abstract

**Aims:**

To investigate the effect of injectable salvia polyphenolic acid on the improvement of limb movement and cognitive dysfunction in acute stroke patients.

**Materials and Methods:**

The clinical data of 90 acute stroke patients were collected for retrospective study and divided into 45 cases each in the comparison group and the observation group according to the different treatment methods; using basic treatment + salvianolic acid, the comparison group implemented conventional alteplase and butalbital treatment, and the observation group used injectable salvianolic acid treatment, to observe and compare the clinical efficacy, changes in neurological deficits, cognitive function, and motor function scores before and after treatment in the two groups.

**Results:**

The NIHSS (National Institute of Health stroke scale) score, cerebral infarct volume, NSE (neuron-specific enolase), and S100*β* (A neurotrophic factor) levels were reduced after treatment compared with those before treatment in this group, and the NIHSS score, cerebral infarct volume, NSE, and S100*β* levels in the observation group were lower than those in the comparison group after treatment, and the difference was statistically significant (*P* < 0.05). Compared with the clinical efficacy of the comparison group and the observation group, the treatment effect of the observation group was better than that of the comparison group, and the difference was statistically significant (*P* < 0.05). After treatment, the cognitive function and motor function scores of both groups were significantly improved compared with those before treatment, and the degree of improvement of each score in the observation group was significantly better than that in the comparison group (*P* < 0.05). During the trial, two patients in the comparison group developed a generalized rash and withdrew from the experiment, and the rash subsided after anti-allergic treatment, and no significant adverse events were observed in the remaining participants. There was no statistically significant difference in liver and kidney function and cardiac enzyme test indexes between the two groups of patients at 14 days of treatment (*P* > 0.05).

**Conclusion:**

Danshen polyphenolic acid for injection has definite clinical efficacy in the treatment of acute ischemic stroke, and it can effectively improve cognitive and motor functions and promote neurological recovery in patients with high safety.

## 1. Introduction

Stroke is a cerebral blood circulation disorder with sudden onset in patients with cerebrovascular disease due to various precipitating factors that cause narrowing, occlusion or rupture of intracerebral arteries, resulting in acute cerebral blood circulation disorders and clinical signs and symptoms of transient or permanent cerebral dysfunction [1]. Stroke is divided into ischemic stroke and hemorrhagic stroke [2]. Acute stroke is the most common type of stroke and is characterized by high morbidity, disability, and mortality, with a poor prognosis that seriously affects the quality of life of patients and their families, making timely and effective treatment of acute stroke patients particularly important [3]. Currently, the most important treatment for acute stroke is thrombolysis, which can be divided into intravenous thrombolysis, arterial thrombolysis, and combined arteriovenous thrombolysis, and thrombolysis within 3-6 h is the most effective [4]. Seventy-five percent of acute ischemic stroke patients will have some degree of motor dysfunction and cognitive impairment, which will not only seriously affect the survival quality of patients, but also increase the burden on their families and society [5]. There are not many effective therapeutic drugs for acute ischemic stroke, and there is a lack of effective preventive measures and drugs for prevention [6]. Salvia polyphenolic acid for injection is mainly an herbal preparation made from the water-soluble extract of Salvia miltiorrhiza, which has certain anti-lipid peroxidation and free radical scavenging effects on brain microsomes [7]. It can increase superoxide dismutase activity and regulate nitric oxide synthase activity, which can protect brain tissues and improve microcirculation, and it has been widely used clinically in the treatment of cerebrovascular diseases with injectable salvia polyphenolic acid [8]. In this study, we intend to observe the effect of injectable salvia polyphenolic acid on the improvement of limb movement and cognitive dysfunction in patients with acute stroke, to provide relevant clinical guidance.

## 2. Material and Methods

### 2.1. Research Object

In this study, 90 acute stroke patients who met the inclusion and exclusion criteria and were admitted to the Department of Neurology of our hospital from January 2020 to January 2022 were selected using a retrospective study method. The diagnosis of acute stroke met the diagnostic criteria in the Chinese Guidelines for the Diagnosis and Treatment of Acute Stroke 2018 [9]: chest pain lasting more than 20 minutes, the presence of diagnostic *Q* waves in a series of ECG recordings, the presence of evolving injury currents lasting more than one day, and at least one of the serum enzyme tests performed within 72 hours of symptom onset or hospitalization that was more than twice the upper limit of normal.

### 2.2. Exclusion Criteria

Inclusion criteria are as follows: (i) age 18-80 years; (ii) all patients in this study had their first onset and received treatment within 6 h; and (iii) intracranial hemorrhage was excluded by cranial CT or magnetic resonance imaging, and there were no early large cerebral infarction imaging changes. Brain CT scans can generally be performed from the base of the skull to the top of the skull, mainly to observe the abnormal density shadows in the brain parenchyma, whether there is cerebral infarction, cerebral hemorrhage or space occupying in the brain. The bone of the base, the fine structure, the resolution is relatively clear, the vestibular aqueduct and the cochlea can be found, or some other structures, such as some temporal bones, sphenoid bones, optic canal, nasal bones, these fine anatomy can be obtained through the skull base CT Even three-dimensional CT of the skull base can be observed. Exclusion criteria are as follows: (i) previous history of intracranial hemorrhage, pregnant and lactating women, and those with contraindications to thrombolysis; (ii) combined with severe cardiac, hepatic, and renal insufficiency; and (iii) those with a history of epilepsy, those with allergy to the drugs treated in this study, and those who have recently taken oral anticoagulants.

## 3. Methods

All patients were given conventional treatments such as oxygenation, improvement of cerebral metabolism, and nerve nutrition, as well as oral atorvastatin (Pfizer Pharmaceutical Co., Ltd., State Drug Administration: H20051408) 20 mg/d and aspirin enteric dissolved tablets (Bayer Healthcare Ltd., State Drug Administration: J20130078) 100 mg/d. The comparison group was given alteplase and butalbital on this basis, namely, alteplase (Boehringer Ingelheim Pharma Gmb H&Co. KG, S20160054) 50 mg intravenous thrombolytic therapy, giving 5 mg alteplase in 1 min intravenous push (China Enbep Pharmaceutical Co., Ltd, State Drug quantification: H20050299) 100 ml intravenous drip, infusion time need to be greater than 50 min, bid, for 2 weeks, and at the same time apply butyl phthalein (State Pharmacopoeia H20050298) orally on an empty stomach, 0.2 g once, four times a day, for 2 weeks.

### 3.1. Observation Indicators

The NIHSS score was reduced by 20%-49%; effective was partial self-care, symptoms basically disappeared, NIHSS score reduced by 50%-89%; basic recovery was complete self-care, symptoms basically disappeared, NIHSS score reduced by ≥90%. Neurological function: Patients were assessed for neurological impairment by comparing NIHSS score, cerebral infarct volume, NSE, and S100*β*. The total score of the NIHSS scale was 42, ≤4 for light stroke and ≥21 for severe stroke, including various aspects such as level of consciousness, gaze, upper and lower limb movement, sensation, and speech [10]. Patients in both groups underwent cranial CT plain scan before and after 2 weeks of treatment to observe the area of cerebral infarction, respectively. Before and after treatment, 5 ml of fasting venous blood was drawn from the comparison group and the observation group, respectively, and the upper serum was collected after centrifugation at 3000 r/min, and serum neuron specific enolase (NSE) and S100*β* protein levels were determined by applying enzyme-linked immunosorbent assay. Cognitive function was assessed using the Montreal Cognitive Assessment (MoCA); the higher the score, the better the cognitive function): Motor function was assessed using the Barthel Index (Barthel): the higher the score, the better the patient's daily motor function.

### 3.2. Statistical Analysis

All statistical data in this study were entered into excel software by the first author and the corresponding author, respectively, and the statistical processing software was SPSS25.0 for calculation. Repeated measures analysis of variance between groups was used to measure the measurement expressed as mean ± standard deviation (X ± S). Count data expressed as a percentage (%) were tested by *χ*2. Univariate and logistic multivariate regression analysis was used to compare the influencing factors, and the risk factors with significant differences were screened. Included data that did not conform to a normal distribution was described by M(QR), using the Mann–Whitney test. All statistical tests were two-sided probability tests. The statistical significance was *P* < 0.05.

## 4. Results

### 4.1. General Information Comparison

In order to study the individual influencing factors of the comparison group and the control group, we classified and counted their general data. The differences were not statistically significant (*P* > 0.05) when comparing the general data of gender, age, BMI, education level, infarct site, disease duration, and combined underlying diseases between the comparison and observation groups, as shown in Table 1.

### 4.2. Comparison of Neurological Function between the Two Groups

There was no statistically significant difference in NIHSS score, cerebral infarct volume, NSE, and S100*β* levels between the two groups before treatment (*P* > 0.05). After treatment, NIHSS score, cerebral infarct volume, NSE, and S100*β* levels were reduced compared with those before treatment in this group, and NIHSS score, cerebral infarct volume, NSE, and S100*β* levels in the observation group were lower than those in the comparison group after treatment, and the differences were statistically significant (*P* < 0.05). This indicates the effectiveness of the treatment regimen (see Figure 1).

### 4.3. Comparison of Cognitive and Motor Function Scores

There was no significant difference in the cognitive and motor function scores between the two groups before treatment (*P* > 0.05), and the cognitive and motor function scores in both groups improved significantly after treatment compared with those before treatment, and the improvement in each score in the observation group was significantly better than that in the comparison group (*P* < 0.05) (see Figure 2).

### 4.4. Safety-Related Indicators

During the trial, two patients in the comparison group developed a generalized rash and withdrew from the experiment, and the rash subsided after anti-allergic treatment; the remaining participants did not see any significant adverse events. There was no statistically significant difference in liver and kidney function and cardiac enzyme test indexes between the two groups of patients at 14 *d* of treatment (*P* > 0.05) (see Figure 3).

### 4.5. The Clinical Efficacy of the Two Groups

Compared with the clinical efficacy of the observation group, the treatment effect of the observation group was better than that of the control group, and the difference was statistically significant (*P* < 0.05) (see Figure 4).

## 5. Discussion

The purpose of this study was to observe the improvement effect of salvianolic acid for injection on limb motor and cognitive dysfunction in patients with acute stroke, in order to provide relevant clinical guidance.

Traditional Chinese medicine has the therapeutic advantages of multiple pathways, links, targets, and components over common Western medicines [10–12]. Danshen polyphenolic acid for injection is extracted from Salvia miltiorrhiza and has a complex composition, which is the best combination of therapeutic effects obtained by numerous pharmacologists after research, and has been found by many scholars to have clear pharmacological effects on cerebral infarction [13]. The quality control of the production process of this drug is carried out from three aspects: cultivation, extraction, and freeze-drying of Salvia miltiorrhiza, and advanced process technology is used to fix the ratio of the content of the active ingredients in the drug to ensure the stability of the components in the drug, which ensures good therapeutic effects and no significant adverse reactions, and provides direction for the treatment of patients with acute ischemic stroke [14, 15].

In our study, the cognitive and motor function scores of both groups improved significantly after treatment compared with those before treatment, and the degree of improvement of each score in the observation group was significantly better than that in the comparison group. Salvia polyphenolic acid for injection belongs to the new class 5 drug of Chinese medicine for injection, which is different from Salvia polyphenolic acid salt preparation, and salvianolic acid is the main active ingredient of Salvia polyphenolic acid for injection, which is a water-soluble phenolic acid component and has the highest content in Salvia [16]. It not only protects endothelial cells and the blood-brain barrier, but also scavenges free radicals and acts as an antioxidant, as well as anti-atherosclerosis, inhibits apoptosis, and effectively protects neural cells [17–19].

This study showed that NIHSS score, cerebral infarct volume, NSE, and S100*β* were all lower in both groups after treatment compared to before treatment in this group, and the difference was statistically significant when the observation group was lower than the comparison group after treatment. NIHSS score scale is the National Institutes of Health Stroke Scale, which is used to assess the degree of neurological deficit after a patient has suffered a cerebral infarction [20]. During the development of acute cerebral infarction disease can cause ischemic and hypoxic damage to brain tissue, leading to rupture of glial cells, and S100*β* protein in the cytoplasm and NSE in neurons are markers of glial cells [21]. Some scholars have shown that the process of acute cerebral infarction causes a large release of NSE and S100*β*, which are present in large quantities in nerves and their secretory other tissues and are released in large quantities into the blood when they are damaged, and S100*β*, which is present in the cytoplasm and has a nutritive effect on neurons, can release large amounts of neurotoxins when they are damaged, so both can be assessed to some extent in terms of neurological impairment The degree of neurological impairment can be assessed to some extent [22–24]. Wang Hongzhi et al. showed that in patients with acute ischemic cerebral infarction, serum S100*β* protein, NSE levels were positively correlated with the degree of neurological impairment [25], and Chu Honggao et al. showed that NIHSS scores and CRP levels were lower after 7 and 15 days of treatment than before treatment, and the observed group of Danshen polyphenolic acid was lower than the group of Danshen polyphenolic acid alone [26]. This study also showed that NIHSS score, cerebral infarct volume, NSE, and S100*β* were lower after treatment compared with the pretreatment period in this group and the differences were statistically significant in the NIHSS score, cerebral infarct volume, NSE, and S100*β* levels after salvianolic acid treatment was lower than those in the comparison group. The results suggest that the treatment of acute stroke with salvia polyphenolic acid is more effective in reducing the degree of neurological impairment of brain tissue in patients than salvia polyphenolic acid alone.

During our study, two patients in the comparison group withdrew from the trial with a generalized rash, which subsided after anti-allergic treatment. After treatment, the cognitive function and motor function scores of both groups were significantly improved compared with those before treatment, and the degree of improvement of each score in the observation group was significantly better than that in the comparison group (*P* < 0.05). During the trial, two patients in the comparison group developed a generalized rash and withdrew from the experiment, and the rash subsided after anti-allergic treatment, and no significant adverse events were observed in the remaining participants. There was no statistically significant difference in liver and kidney function and cardiac enzyme test indexes between the two groups of patients at 14 days of treatment (*P* > 0.05). There were no statistically significant differences in liver and kidney function and cardiac enzyme test indexes between the two groups of patients at 14 days of treatment. In this study, it was found that the degree of neurological deficits improved in both groups after treatment and the improvement was more pronounced in the observation group, with a greater proportion of patients with a good prognosis and a smaller proportion of patients with a poor prognosis, indicating that the use of injectable salvianolic acid was an independent predictor of good prognosis after acute ischemic stroke patients [27]. This indicates that both the observation and control groups were effective in the treatment of acute cerebral infarction patients with clinical prognosis, but the effect was more pronounced in the observation group [28]. Also, no clear drug-related adverse reactions of liver, kidney, and cardiac enzyme abnormalities and other adverse events occurred during this study, suggesting good effectiveness of injectable salvianolic acid in the treatment of acute ischemic stroke, as well as providing a drug option for patients with acute ischemic stroke combined with liver, kidney, and cardiac insufficiency [29].

The present study is a clinical trial study with many confounding factors, which may affect the results, for example, some patients have combined butalbital or erythromycin, and although the dosing is balanced between the two groups, the combined dosing may have an effect on the therapeutic effect, which needs further study. In conclusion, the treatment of acute ischemic stroke with injectable salvianolic acid has definite clinical efficacy, and it can effectively improve the cognitive and motor functions of patients and promote the recovery of neurological functions with high safety. In the future, we will focus on the controversies in the treatment of acute ischemic stroke with salvianolic acid for injection, and increasing the sample size will make the research results more convincing. At the same time, the proportion of severe stroke should be increased, and the influence of more external factors should be considered, so as to minimize the influence of the therapeutic effect caused by the combined administration and ensure the reliability of the results and the safety of salvianolic acid for injection.

## Figures and Tables

**Figure 1:** Comparison of neurological function between the two groups; all nerve function data in our study were entered into excel software by the first author and the corresponding author, respectively, and expressed as mean ± standard deviation. There was no significant difference in infarct volume, NSE, and S100*β* levels (*P* > 0.05). After treatment, the NIHSS score, cerebral infarction volume, NSE, and S100*β* levels in the group were all decreased compared with those before treatment, and the NIHSS score, cerebral infarction volume, NSE, and S100*β* levels in the observation group after treatment were lower than those in the control group after treatment, and the differences were statistically significant. Significance (*P* < 0.05).

**Figure 2:** Comparison of tumor marker levels. All the comparisons of cognitive and motor function scores data in our study were entered into excel software by the first author and the corresponding author, respectively, and expressed as mean ± standard deviation. There was no significant difference in the scores of cognitive function and motor function before treatment (*P* > 0.05), the scores of cognitive function and motor function in the two groups after treatment were significantly improved compared with those before treatment, and the improvement of each score in the observation group was significantly better than that in the control group (*P* > 0.05).

**Figure 3:** Comparison of tumor marker levels. All safety-related index data in our study were entered into excel software by the first author and the corresponding author, respectively, and expressed as mean ± standard deviation. The statistical processing software was SPSS25.0 for calculation and chi-square test. The patient with systemic rash was withdrawn from the experiment, and the rash subsided after anti-allergic treatment, and the remaining participants had no obvious adverse events. There was no significant difference in liver and kidney function and myocardial enzyme detection indexes between the two groups on the 14th day of treatment (*P* > 0.05).

**Figure 4:** The clinical efficacy of the two groups. All the data of our study were entered into excel software by the first author and the corresponding author, respectively, represented by integers, and the statistical processing software was SPSS25.0 for calculation. The chi-square test was used to find that the clinical efficacy of the control group was compared with that of the observation group. The effect was better than that of the control group, and the difference was statistically significant (*P* < 0.05).

**Table 1:** Comparison of general information between two groups of patients.

Normal information	Comparison group (45)	Observation group (45)	*t*/*χ*^2^	*P*
Gender				
Male	21	26	1.113	0.291
Female	24	19		
Age	58.30 ± 12.40	59.00 ± 11.80	0.274	0.784
BMI (kg/m^2^)	22.73 ± 3.25	23.15 ± 3.43	0.596	0.553
Educational level				
Junior high school and below	15	15	0.884	0.643
High school or secondary school	25	22		
College and above	5	8		
Infarct site				
Base	18	17	0.377	0.828
Brain stem	20	18		
Cerebellum	17	20		
Time from onset to admission (min)	160.02 ± 23.64	163.25 ± 22.52	0.664	0.509
Combined underlying diseases Normal information Gender				
Hypertension	5	8	0.819	0.664
Diabetes	19	18		
Coronary heart disease	21	19		

## Data Availability

The experimental data used to support the findings of this study are available from the corresponding author upon request.
